This article has been retracted.

# Public Security Video Image Detection System Construction Platform in Cloud Computing Environment

**DOI:** 10.1155/2022/4113803

**Published:** 2022-02-10

**Authors:** Hexiao Yin

**Affiliations:** School of Criminal Law, East China University of Political Science and Law, Shanghai 201620, China

## Abstract

The public security image detection system is an important way to assist the police in the investigation. In today's cloud computing environment, the processing power of cloud computing is gradually improving. In order to explore its application in the investigation system, this paper constructs a public security video image investigation system based on cloud computing environment. This paper uses cloud computing technology to improve the processing capacity of the system. It then combines the storage capabilities of the backend server implementation technology and the working principle of Hadoop to construct a basic model. Then combined with the storage capability of the backend server implementation technology and the working principle of Hadoop and CP-ABE encryption, decryption, and reconstruction, a basic model is constructed. This paper also designs public security video surveillance system vehicle detection and test experiments, cloud storage encryption algorithm experiments, and computational storage requirements analysis experiments. It optimizes the system based on the results of the experiment and finally compares it with the traditional investigation system. The experimental results show that the public security video image detection system based on cloud computing can improve the accuracy by 5%–25% compared with the traditional detection system. And the public security video image detection system based on cloud computing can increase the efficiency by 2%–17% compared with the traditional detection system.

## 1. Introduction

In order to maintain long-term social stability, the Ministry of Public Security launched the National Ministry of Public Security's strong police demonstration city construction project to strengthen urban construction and science and technology. Major cities across the country have launched large-scale scientific and safe urban governance programs. At two meetings in 2017, the government proposed to strengthen the integration of police operations and the Internet in order to improve the efficiency of public security operations.

In recent years, with the active advancement of the construction of the “Skynet” video surveillance project, it has played an increasingly important role in maintaining social order, preventing street crimes, ensuring public safety, and responding to emergencies. Incidents caused by its insufficient investigative capabilities are also increasing, which also highlights the lack of domestic video image investigative capabilities [1].

Mobile users usually have a high demand for localized and location-based information services [2]. Deng et al. expand cloud computing by deploying localized computing facilities on the premise of users and prestore and distribute cloud data to mobile users with fast local connections [3]. They are researching fog computing to expand cloud computing capabilities and storing and distributing operational data to users, but they have few applications in public safety video image detection systems. The existing static grid resource scheduling algorithms are limited to minimizing the completion time and cannot meet the requirements of cloud computing for resource scheduling. Wei et al. proposed a cloud resource allocation model using Hidden Markov Model (HMM) in a cloud computing environment based on the incomplete information Stackelberg game (CSAM-IISG) [4]. Their research is mainly based on the use of hidden Markov Models in the cloud computing environment. Although it is not related to the investigation system, there are still many places to refer to. Data sharing has become an attractive service provided by cloud computing platforms due to its convenience and economy. Jin et al. solved this challenging problem by proposing a new attribute-based data sharing scheme, which is suitable for mobile users with limited resources in cloud computing [5]. The main purpose of the study by Jin et al. is to solve the problem of data sharing. Therefore, the research is based on cloud computing, and if it can involve public security investigation work, it will be of great help to this paper. Encryption based on password policy attributes (CP-ABE) is always the recommended encryption technology to solve the problem of cloud computing secure data sharing. Wang et al. proposed an efficient cloud computing encryption scheme based on file-level attributes. After they merge the hierarchical access structure into a single access structure, they use a comprehensive access structure to encrypt hierarchical files [6]. Their main research is the encryption problem of cloud computing. If cloud computing can be applied to video surveillance, it will be more in line with the purpose of this paper. In order to study D2D-based public safety video sharing solutions, Zhao et al. studied focal geographic area (FGA) video composed of multiple camera streams. Its bandwidth consumption is higher than that of traditional single-camera streaming, which attracts a large number of content delivery requests in emergency situations [7]. The article by Zhao et al. is mainly based on the application of D2D in public safety video to improve the coverage area of the investigation system and on cloud computing. Video applications are considered an important and important service of the national public safety broadband network. Budny et al.'s contribution to meeting this need is the first to use open source technology to demonstrate how to conduct video experiments in the FirstNet Innovation and Test Lab. They transmit videos from datasets through public safety and commercial broadband networks and under different network conditions [8]. With the installation of a large number of public safety and traffic infrastructure cameras, video analysis has become an important part of public safety [9, 10]. It is impractical to analyze large-scale real-time video streams on the cloud. The purpose of Zhang et al.'s study is to provide a glimmer of hope for edge solutions for video analysis on (or close to) cameras [11]. Their purpose also is to conduct video analysis in the context of the cloud, which is mostly the same as the subject of this paper. It can refer to the application of cloud computing in video analysis. In cloud computing, massively parallel distributed processing services are provided, in which a huge task is split into multiple subtasks, and these subtasks are processed on clusters of machines called workers [12]. Hirai et al. model the task scheduling server as a single-server queue, where the server is composed of many workers [13]. They mainly research task scheduling servers in the context of local cloud computing, and they do not involve much in public security video surveillance work.

The innovation of this paper lies in the use of cloud computing technology, backend server implementation technology, and Hadoop working principles, combined with pedestrian-related knowledge elements in the video data of the video image detection system and public safety video image information. It preprocesses the image to improve the accuracy and efficiency of image acquisition.

## 2. Designing Public Security Investigation System Based on Cloud Computing

### 2.1. Cloud Computing Technology

Matter, energy, information, our food, clothing, shelter, and transportation are inseparable from the support of matter. The development of all things in human life is due to the existence of energy. Cloud computing is now used in various fields, especially in developers with more convenient and flexible applications [14, 15]. Demanders can use them as needed, calculate the services they need, and then purchase them as planned, without causing waste. Users purchase the resources they need at a lower cost through computing and service models, just like people buying water, electricity, and gas in their daily lives.  Figure 1 shows the application block diagram of cloud computing.

At present, cloud computing early warning has spread to all aspects of our lives: when enjoying the fast shopping on Taobao, cloud computing technology has provided a powerful impetus for hundreds of millions of transactions; when using 12306 to purchase tickets, cloud computing technology [16] escorted hundreds of millions of ticket purchase requests; when using QQ WeChat chat, cloud computing technology provides services for massive data exchange information. In 2016, Alibaba Cloud collaborated with more than 500 large enterprises to launch cloud computing solutions. At present, cloud computing technology has shifted from small projects (such as games, mobile, and e-commerce) to large projects [17] (such as transportation, finance, and government). In 2016, Tencent Cloud provided more than 10 cloud servers, which were also officially launched in data centers in Western countries such as Europe, and many large and small companies have also applied cloud computing technology to their own development. It can be seen that the development of cloud computing technology is increasing day by day, and it will become more and more popular [18]. The three business models of cloud computing are shown in Figure 2.

As shown in the figure, there are three business models for cloud servers: IaaS model [19] (architecture services), PaaS model [20] (platform services), and SaaS model [21] (software services). In order to make the online work run smoothly, the IaaS model provides server, storage, network, and operating system services. Enterprises use this model to build cloud computing management platform and server virtualization software development; the PaaS model mainly provides a development service platform, which can provide fast and efficient services for coding and deploying applications. This model mainly does the following tasks: service establishment, cloud platform management, data security maintenance, and performance optimization; the SaaS model provides users with software application services through the network. Enterprises in this mode are mainly engaged in the following tasks: cloud application software development, sales of cloud computing management platforms, and cloud application software systems.

#### 2.1.1. Backend Server Implementation Technology

This system is based on a cloud server system, and users use a browser to interact with a background server. The system is divided into web server, RTMP video streaming server, and database server. The web server uses the Tomcat server conforming to the JavaEE specification to construct the service framework and business logic; the RTMP video stream server uses the Nginx RTMP module to provide video stream distribution; the database server uses the nonrelational database MongoDB to store real-time sensor data.

Java Enterprise Specification (J2EE) [22] is a technology platform developed by Sun [23] for large-scale company-level web server backend service programs using Java language. Sun hopes to use this to standardize enterprise-level application development. The proposal of standard reusable modular components and the automatic processing of project construction have greatly simplified the development of application programs and at the same time reduced the requirements for programming and trained programmers.

Large-scale company-level projects are more flexible, expandable, and easy to maintain after being built using J2EE technology.

*(1) Keep Existing IT Assets*. Because of the fierce market competition, companies must always adapt to new market demands. It is important to use the existing project organization structure to realize new market demand functions and to avoid overthrowing the existing structure and reformulating the project structure plan.

*(2) Efficient Development*. J2EE enables project developers to focus more time and energy on developing business logic. Some general, repetitive, and cumbersome background basic logic is handed over to the corresponding middleware vendors to complete, which shortens the development time.

*(3) Unlimited Operating Environment*. J2EE makes it possible to develop certain programs that need to run in a heterogeneous environment. J2EE-based application projects do not need to rely on any specific software system or specific hardware system.

*(4) Scalability*. In order to meet the increasing number of customers using the company's platform, companies need to choose a server-side platform with high scalability. Company projects based on the J2EE platform have a wide choice of server-side platforms due to the characteristics of J2EE's unlimited operating environment.

*(5) Stable Availability*. The server-side platform must meet the needs of 7 × 24 hours operation due to the characteristics of Internet applications. If the server shuts down unexpectedly, it will cause catastrophic loss of user data.

In the intelligent video surveillance system, the accuracy of the video image recognition algorithm is largely affected by the video image quality of the network video stream. The transmission bandwidth, real-time performance, and definition of video images are high, so high requirements are put forward for the transmission of video streams. So this system uses RTMP protocol to transmit real-time data. The server uses OpenCV's built-in FFMPEG to analyze RTMP protocol data, and after decoding, it is analyzed by the image recognition algorithm, and the result is fed back to the web server. After the web server gets the result, it pushes the result to the user.

#### 2.1.2. Hadoop Working Principle

In distributed storage and computing, Chen et al. [24] used a master/slave architecture to run Hadoop through background programs, which are composed of Job Tracker, Data Nade, Name Node, Task Tracker, and so on. Its core design ideas are MapReduce, Zookeeper, and HDFS.

The Hadoop platform can provide three ways of working. Stand-alone mode (default installation mode): all configuration items are empty, and the system runs in stand-alone mode for program development and debugging; pseudodistributed mode: on the basis of single-machine mode, some simple functions such as memory checking, input, and output of distributed operation are added; in fact, all DataNodes run on the same PC and run the Hadoop system in a single node mode; fully distributed mode: it is to form a real Hadoop cluster and run it, install Hadoop on different computers, and connect different computers. It can be clearly seen from the above that, in order to realize the storage and processing of large-scale video data and to realize real-time monitoring and calling of video conditions in various places and fields, we need to build a distributed cluster in a fully distributed mode.

HDFS [25] reads and processes large files by accessing data streams and has the functions of automatic detection, automatic repair, and data backup. It mainly adopts a master-slave structure mode, and a cluster includes a master node (master) and multiple DataNodes (slave). It is shown in Figure 3.

### 2.2. Video Image Detection System

The powerful video image detection function [26] helps prevent the occurrence of criminal cases. Video image survey is a combination of the latest computer technology, video collection technology, network transmission technology, and big data technology. The video image detection function is very important to maintain public security and social stability, and it will indeed play a greater role in the new historical era.  Figure 4 shows the structure of the video image detection system.

Video image investigation presents objective facts in front of investigators in the form of videos and photos. Investigators can use the intuitiveness of video and images to perform the same identification, tracking, and discovery of clues to related events.

#### 2.2.1. Pedestrian-Related Knowledge Elements in Video Data

In order to better describe the pedestrian status information in different surveillance scenarios, the comprehensive analysis of pedestrians in the video big data environment can be realized. It needs to abstractly describe the scenes involved in the analysis of pedestrian behavior in video surveillance and some information of pedestrians based on the knowledge metamodel [27]. The basic knowledge element includes environmental knowledge element, surveillance camera knowledge element, scene knowledge element, event knowledge element, behavior knowledge element, pedestrian knowledge element, and relationship knowledge element. Pedestrian knowledge elements can be subdivided into single knowledge elements and crowd knowledge elements. The relational knowledge element is mainly used to describe the relationship between the basic knowledge elements and the relationship between the attributes of the basic knowledge elements.

*(1) Environmental Knowledge Element*. The environment, also called weather, is the change in the state of the atmosphere within a certain time interval. The state of the weather will affect the apparent state of things to a certain extent. For example, the behavior habits and behaviors of pedestrians are different under clear weather and rainy and snowy weather. At the same time, the weather state and light intensity will also affect the actual state and imaging conditions of objectively existing things in the monitoring scene and then affect the accuracy of the video processing algorithm. Therefore, it is necessary to define environmental knowledge elements.

*(2) Surveillance Camera Knowledge Element*. The video surveillance system mainly includes front-end camera part, transmission part, control part, display part, power supply system, and antitheft alarm part.

*(3) Scene Knowledge Element*. For a specific monitoring scene, fixed things such as trees, buildings, and street lights in the scene are called objectively existing things. First, the background image of the scene is acquired based on the surveillance camera, and then the segmentation state of the background image is obtained according to the image segmentation algorithm in the operator library. It combines the scene segmentation state with the foreground extracted from the recorded video, which can effectively eliminate the influence of noise on the video processing accuracy and processing speed. That is, in the process of video image processing, only the scene area where pedestrians may exist is considered, which can improve the accuracy and extraction speed of foreground pedestrian primitives.

*(4) Event Knowledge Element*. According to the survey results, the social security emergency management based on the video surveillance system mainly focuses on the following events in the surveillance scenario: border intrusion incidents, cross-line detection incidents, wandering detection incidents, population statistics, crowd gatherings, stampede incidents, violent incidents, crowd fights, and other incidents.

*(5) Behavioral Knowledge Elements*. The behavioral knowledge element is mainly based on the pedestrian behavior image library, and the common feature representation is based on the knowledge discovery for different behavior categories in the common sense knowledge.

*(6) Video Knowledge Element*. Video knowledge element is mainly used to record the main information of video clips. There are many tools for recording video, such as mobile phones, video recorders, tablets, computers, and surveillance cameras.

#### 2.2.2. Public Safety Video Image Information

Public safety video image information [28] is to maintain public safety, and administrative agencies use video image acquisition equipment to produce or obtain video image information about public safety places and areas. It is the extensive construction and in-depth application of this system by administrative agencies. Video images continue to meet the information needs of government management and social services, but the disclosure of this information also triggers the risk of infringement of civil rights.

Public safety video image information has the following characteristics.

First, the purpose is to safeguard the public interest. Obtaining video image information is a means, and maintaining public safety is the goal. Public safety involves factors that affect social safety such as theft and robbery and factors that affect traffic safety such as speeding and retrograde. Video image information is used in various fields of public security, which improves the government's management and service efficiency. Factors that affect food safety include illegal production and processing, forest fires, etc., that affect fire safety, and even factors that involve environmental monitoring and other fields.

Second, the collection area is a public space. There is no need for a specific majority of people to enter freely, and the space is open. Video image acquisition equipment is installed in public areas such as streets, stations, squares, and vital parts, which is completely open. There are also public places in specific areas such as communities or campuses, libraries, bank business halls, shopping malls, subways, and buses, which are semiopen. It does not include personal spaces such as homes and dormitories.

Third, the content is comprehensive. Different from ordinary government information disclosure in the form of text, pictures, and so on, a video image is a collection of data information. As long as it enters the video shooting range, all behaviors and activities of the parties will be objectively and comprehensively recorded. The content contains various information such as appearance, sound, and action, which provides the viewer with more direct sensory stimulation in visual and auditory sense, and is complex and real-time. For example, the whole law enforcement process of the seizure and seizure of law enforcement officers captured by the law enforcement recorder is a collection of a series of information, including the appearance, voice, and actions of the law enforcement officers and the parties.

Fourth, the collection equipment is diversified. With reference to the State Council's guidance on the implementation of the whole-process recording system for law enforcement, a variety of video image capture devices are listed. The acquisition equipment is mainly fixed video equipment, supplemented by mobile equipment such as body cameras and cameras. With the deep integration of technology, new types of equipment such as drones adapt to meet the needs of different scenarios, and video equipment becomes more intelligent. The video collection methods range from a single collection method of fixed video equipment to a variety of collection methods such as body enforcement recorders and drones.

Fifth, the management subject is statutory. The main body includes both the main body that records the video and the main body that obtains the video from other places according to law, mainly including the public security department, the national security department, the transportation management department, the fire safety management department, and other administrative bodies. In practice, public security organs are used as competent departments to build video and image information network sharing platforms in many places. Its grasp of the video information is more comprehensive, and the disputes are mostly concentrated in the department, so this paper focuses on the discussion of the public security organ's video image information disclosure scope.

### 2.3. Image Preprocessing

#### 2.3.1. Homomorphic Filtering

Homomorphic filtering [29] is a combination of grayscale conversion and frequency domain filtering, which can improve contrast and achieve grayscale stretching at the same time. The basic flow of the algorithm is as follows:

(1) First, the original image *f*(*a*, *b*) is regarded as the product of illuminance and reflection [30]. Here, *p*(*a*, *b*) is the illuminance and *s*(*a*, *b*) is the reflection component.
  (1) $$\begin{array}{c} f\left(a,b\right)=p\left(a,b\right)\cdot s\left(a,b\right). \end{array}$$
(2) First, it performs a logarithmic transformation on both sides of formula (1) to separate the two parts of illuminance and reflection.
  (2) $$\begin{array}{c} \ln\left(f\left(a,b\right)\right)=\ln\left(p\left(a,b\right)\right)+\ln\left(s\left(a,b\right)\right). \end{array}$$
(3) It performs Fourier transform on both sides of formula (2), converts to frequency domain, and obtains the following equation:
  (3) $$\begin{array}{c} F\left(x,y\right)=P\left(x,y\right)+S\left(x,y\right). \end{array}$$
(4) Using a filter processing with a transfer function of, let
  (4) $$\begin{array}{c} C\left(x,y\right)=G\left(x,y\right)F\left(x,y\right)=G\left(x,y\right)P\left(x,y\right)+G\left(x,y\right)S\left(x,y\right). \end{array}$$
(5) It performs the inverse Fourier transform [31] of the filtering result of the previous step and converts it into the time domain.
  (5) $$\begin{array}{c} c\left(x,y\right)=\gamma^{-1}\left\{C\left(x,y\right)\right\}=p\left(a,b\right)+s\left(a,b\right). \end{array}$$
(6) The pair performs an exponential operation to obtain an enhanced image.
  (6) $$\begin{array}{c} h\left(x,y\right)=q^{c\left(x,y\right)}=q^{p^{\prime }\left(a,b\right)}q^{s^{\prime }\left(a,b\right)}. \end{array}$$

It can be seen from the above algorithm flow that the most important thing in quasi-identical filtering is the selection of filters. The form of the quasi-identical filter used in this paper is as follows:

(7) $$\begin{array}{c} G\left(x,y\right)=\left(s_{g}-s_{I}\right)\left(1-\exp\left[-c\cdot \frac{T^{2}\left(x,y\right)}{T_{0}^{2}}\right]\right)+s_{I}. \end{array}$$

Among them, *s*_*I*_ and *s*_*g*_ are adjustment parameters (*s*_*I*_ < 1, *s*_*g*_ > 1), and *z* is a constant, which controls the clarity of the filter function. *T*(*x*, *y*) is the distance between point (*x*, *y*) and the center frequency point (*U*, *V*), and *T*_0_ is the variance of the Gaussian function [32].

(8) $$\begin{array}{c} T\left(x,y\right)={\left[{\left(x-\frac{U}{2}\right)}^{2}+{\left(y-V/2\right)}^{2}\right]}^{0.5}. \end{array}$$

#### 2.3.2. Retinex

As shown in Figure 5, the incident light illuminates the object S for diffuse reflection, and the reflected light finally forms an image at the observation end.

(9) $$\begin{array}{c} E\left(a,b\right)=S\left(a,b\right)\cdot I\left(a,b\right). \end{array}$$

It uses a low-pass filter [33] *F*(*a*, *b*) and convolution of the original image to obtain low-frequency information.

(10) $$\begin{array}{c} \log\;S\left(a,b\right)=\log\frac{S\left(a,b\right)}{I\left(a,b\right)}\\ =\log\;S\left(a,b\right)-\log\left(F\left(a,b\right)*S\left(a,b\right)\right). \end{array}$$

Among them, *F*(*a*, *b*) is the Gaussian convolution function.

(11) $$\begin{array}{c} F\left(a,b\right)=\phi \cdot \;\exp\left(\frac{-\left(a^{2}+b^{2}\right)}{z^{2}}\right), \end{array}$$

where *φ* is a constant matrix, which satisfies

(12) $$\begin{array}{c} \iint F\left(a,b\right)da\text{d}b=1. \end{array}$$

The MSR algorithm ensures the enhancement of details and the fidelity of colors. The formula is as follows:

(13) $$\begin{array}{c} \log\;S\left(a,b\right)=\sum_{n=1}^{N}W_{n}\left\{\log\;I_{l}\left(a,b\right)-\log\left(F\left(a,b\right)*S\left(a,b\right)\right)\right\},\;l=1\ldots K, \end{array}$$

where *W*_*n*_ represents SSR of different scales for weighting *l* is the color channel, and generally *K* = 3 (*R*, *G*, *B* three channels).

#### 2.3.3. Smooth Linear Filtering

Smooth linear filtering [34] is a general term for many spatial filtering methods, as shown in Figure 6; the most commonly used are four neighbors and eight neighbors.

*(1) General Threshold*. The general threshold value is the best threshold value line by line proposed in 1994, and it is also the most commonly used and simplest threshold value. The selection criteria are as follows:

(14) $$\begin{array}{c} \mu =\theta_{k}\sqrt{x\;\ln\;K}. \end{array}$$

*(2) Bayesian Shrinkage Threshold*. In the Bayesian framework, the Bayesian shrinkage threshold is achieved by minimizing the Bayesian risk.

(15) $$\begin{array}{c} \mu =\frac{\theta_{K}^{2}}{\theta_{a}}. \end{array}$$

Among them, *θ*_*K*_^2^ is the variance of the noise, and *θ*_*a*_ is the standard deviation of the wavelet coefficients in the subband, which can be estimated using the following formula:

(16) $$\begin{array}{c} \theta_{a}=\sqrt{\max\left(\theta_{s}^{2}-\theta_{K}^{2},0\right)}. \end{array}$$

Among them,

(17) $$\begin{array}{c} \theta_{s}^{2}=\frac{1}{K}\sum_{i=1}^{K}b{\left(i\right)}^{2}. \end{array}$$

So the noise model of the image is

(18) $$\begin{array}{c} x_{0}\left(a,b\right)=x\left(a,b\right)+y\left(a,b\right). \end{array}$$

Among them, *x*_0_ is the observed image, *x* is the image without noise pollution, and *y* is Gaussian noise with 0 noise and *θ*^2^ variance.

## 3. Public Safety Video Detection Experiment

### 3.1. Vehicle Detection and Test Experiment of Public Safety Video Surveillance System Based on Cloud Computing

In this experiment, two Linux clusters installed on the rack are used. One is composed of 16 1 GHz Pentium II nodes (each node has 512 MB of memory). Each node runs the Red Hat Linux kernel version 2.4.20-8, and the Java runtime version is J2SDK1.5.006-b05. The other is an Itanium 2 server with 20 dual-core 1.3 GHz. The nodes in the cluster are connected through a 100 Mbps Ethernet switch. The kernel version of each node running Red Hat Linux is 2.4.0-2, the Java runtime version is J2SDK1.5.003-b07, and the two clusters are connected through 100 Mbps bandwidth.

In the following experiment, NonD represents a general maintenance program that does not consider dependencies, such as ProActive and SmartFrog; SRL means maintaining the service in accordance with the shell script sequence; CG-0 means calling a maintenance plan that depends on perception; CG-1 represents the group maintenance plan with feedback; and REQ represents the fixed request rate from the service component.

In order to verify the influence of propagation dependency and deployment dependency, the experiment set the fixed request rate of the request distribution service to 6 requests per second. At 15 seconds, the maintenance program is entered into the running license plate retrieval service. This experiment tested three solutions: NonD, SRL, and CG-0. The next experiment will test the vehicle detection service and set the fixed request rate to 10 requests per second. The result is shown in Figure 7.

As can be seen in the figure, before the maintenance process started, the system was running well, and when the maintenance started in 15 s, the system throughput of the three different schemes all dropped to zero. Although the figure shows that the maintenance process of NonD ended the earliest, the system did not work properly, and finally, the maintenance of the license plate extraction service failed. This is because NonD did not consider the AND dependency between the license plate extraction service and the shape analysis service. Compared with CG-0, although the SRL program successfully completed the system maintenance, it took too much time to affect the availability of the system, and CG-0 achieved relatively high efficiency. Similarly, two different solutions, CG-0 and CG-1, were launched at 15 s. The CG-0 scheme spreads the maintenance tasks to the node virtual machines related to the vehicle detection service, and the entire propagation process takes 62.97 s. However, it can be found from the figure that the amount of swallowing leaves of CG-0 in the execution process is close to zero, and about 57.9% of the requests are lost at the same time. Compared with CG-0, the CG-1 scheme optimizes the dependencies through grouping dependencies and obtains better experimental results. It maintains target services by setting different priorities. As can be seen from Figure 7, the effect of this improvement is obvious. First, the throughput during the maintenance process has increased to 7.08 requests/sec. Although the average response time was 929.8 ms, which was twice that before maintenance, the request loss rate dropped from 57.9% of the CG-0 scheme to 25.6%. At the same time, because the vehicle detection service is a key service of the system, it is difficult to avoid the vehicle detection service according to the execution semantic relationship of the system, and the cost of 25.6% is almost the minimum of *n* solutions.

### 3.2. Cloud Storage Encryption Algorithm Experiment

The user's private key will be associated with any number of attributes represented as strings. When a party encrypts a message, it specifies the associated access structure on the attribute. If a user's attributes are passed through the ciphertext's access structure, the user can only decrypt that ciphertext and handle more complex access controls, such as numeric ranges, by transforming the access tree into a smaller access tree.

Traditionally, this type of access control was implemented by using trusted servers to store data locally. Increasingly, however, data is stored in a distributed fashion across many servers. The downside is that it is increasingly difficult to keep data secure using traditional methods. When data is stored in multiple locations, the chances of one of them being compromised are greatly increased.

In order to verify that the video encryption algorithm in this paper can meet the real-time requirements, the six basic video sequences are packetized, encrypted, decrypted, and reconstructed.  Table 1 shows the increase in encoding and decoding time for different sequences caused by video encryption and decryption operations. From the data in the table, it can be seen that the method of encrypting key data packets in this paper can meet the real-time requirements.

The efficient access policy update method proposed in this paper is to subpackage the video based on data dependency coding and use CP-ABE to encrypt the key data group and upload it to the cloud storage server. When updating the access control policy, the video data owner only needs to retrieve the key data packets from the cloud to decrypt and reencrypt. The update process only involves critical data packages, not critical data packages. It is not affected and can greatly reduce the computational burden and network resource consumption brought by the update process to the video owner and effectively improve the update efficiency of the CP-ABE access control strategy.  Table 2 shows the proportion of key data and nonkey data in six different video sequences when GOP = 15. It can be seen from the table that the key data in the coded video only accounts for a small part of the total video data.

For the same coded video, if the GOP value in video coding changes, the proportion of key data in the total video data will also change accordingly.  Figure 8 shows the relationship between the basic video sequence Football and Flower key data with the GOP value.

It can be seen from the figure that the larger the GOP value, the lower the proportion of key data in the total data. The efficient access control strategy update method proposed in this paper can effectively reduce the amount of data involved in the update process. The more the update times, the more obvious the effect.

Figure 9 shows the amount of encrypted/decrypted data required to update the access control policy for the video sequences Football and Flower under GOP values of 7 and 15, respectively. The size of the original video sequence is set to 100 standard units. It can be seen from the figure that the access control policy update method in this paper is compared to directly adopting CP-ABE encryption and encoding video to realize video sharing applications in the cloud. It can significantly reduce the amount of encrypted and decrypted data required in the video during the update process and reduce the computational burden of the video data owner to update the access control strategy.

The owner of the encoded video data updates the access control policy and needs to download the encrypted encoded video from the cloud. After adjusting the access control policy locally, the encrypted encoded video needs to be reuploaded to the cloud server. Although video files are compressed, the amount of data is generally still large. If the data owner frequently updates the access control strategy, the upload and download process will consume a lot of network resources. The efficient access control policy update method in this chapter can effectively reduce the amount of data encrypted and decrypted by the owner and greatly reduce the consumption of network resources.

## 4. Public Security Investigation System Based on Cloud Computing

### 4.1. Calculation and Storage Requirements

H.264 compression is currently the most effective compression technology. Compared with the 4Part2 standard of M.JPEG and MPEG, the H.264 encoder can reduce the size of digital video files by 80% and 50%, respectively, without affecting the image quality. This means that H.264 files require less bandwidth and storage space.

Tables 3–5 illustrate the storage calculation results of the three compression formats. Because there are many variables that affect the average bit rate, the calculations of H.264 and MPEG-4 are not necessarily very accurate. M.JPEG has an accurate calculation formula because each image of M.JPEG only has one file. The storage requirements of M.JPEG records vary depending on the frame rate, resolution, and compression level.

#### 4.1.1. H.264 Calculation

Approximate bit rate/8 (the number of bits in a byte) × 3600 s = KB per hour/1000 = MB/d, hour.

MB/hour × working hours per day/1000 = GB/day.

GB/day × required storage time = storage demand.

#### 4.1.2. MPEG.4 Calculation

Approximate bit rate/8 (the number of bits in each byte) × 3600 s = KB per hour/1000 = MB/d, hour.

MB/hour × working hours per day/1000 = GB/day.

GB/day × required storage time = storage demand.

*Note*. The formula does not consider exercise flow, which is an important factor that affects the amount of storage required.

#### 4.1.3. M.JPEG Calculation

Image size × frame/second × 3600 s = Kilobyte(1④)/1000 = Megabyte(MB)/d, hour.

MB/hour × working hours per day/1000 = Gigabyte(GB)/day.

GB/ × required storage duration = required storage.

### 4.2. Comparative Experimental Analysis of Public Security Video Image Detection System Based on Cloud Computing and Traditional Detection System

In order to study the advantages and disadvantages of the design of the public security video image detection system based on cloud computing and the traditional detection system, this paper designs a comparison experiment of the accuracy and efficiency of the public security video image detection system based on cloud computing. The experimental results are shown in Figure 10.

It can be seen from the figure that the accuracy of the public security video image detection system based on cloud computing can reach 80%–95%, while the accuracy of the traditional detection system is only 70%–75%. This new type of investigation system has improved the accuracy by 5%–25% compared with the traditional investigation system. And the efficiency of the public security video image detection system based on cloud computing can reach 82%-92, while the efficiency of the traditional detection system is only 75%–80%. Compared with the traditional detection system, the efficiency of the public safety video image detection system based on cloud computing has increased by nearly 2%–17%. This shows that the public security video image detection system based on cloud computing is much higher in accuracy and efficiency than the traditional ones.

## 5. Conclusions

This paper mainly studies the construction of a public security video image detection system platform in a cloud computing environment. This paper uses the processing power of cloud computing technology, the backend storage capability of the backend server implementation technology, and the working principle of Hadoop, combined with pedestrian-related knowledge elements in the video data of the video image detection system and public safety video image information. It preprocesses the image and finally builds a public security video image detection system based on cloud computing.

## Figures and Tables

**Figure 1:** Application block diagram of cloud computing.

**Figure 2:** Three business models of cloud servers.

**Figure 3:** HDFS architecture.

**Figure 4:** Video image detection system structure.

**Figure 5:** Principle of object imaging.

**Figure 6:** Schematic diagram of 4-neighborhood and 8-neighborhood.

**Figure 7:** Results of vehicle detection experiment. (a) Throughput during maintenance of license plate extraction service. (b) Throughput during maintenance of vehicle inspection service.

**Figure 8:** Changes in the proportion of key data in total video data.

**Figure 9:** The amount of encrypted/decrypted data required to update the access control policy. (a) GOP = 7. (b) GOP = 15.

**Figure 10:** Comparison of experimental results. (a) Accuracy comparison. (b) Efficiency comparison.

**Table 1:** Percentage increase in video processing time.

Video sequence	Encoder (%)	Decoder (%)	Total (%)
Bridge	1.83	2.71	4.54
Flower	1.77	2.46	4.23
Stefan	1.49	1.73	3.22
Mobile	1.63	2.10	3.73
Football	1.59	1.84	3.43
Salesman	0.96	2.83	3.79

**Table 2:** Video sequence data ratio when GOP = 15.

Video sequence	Key data (%)	Noncritical data (%)	Total (%)
Bridge	20.48	79.52	100
Flower	17.54	82.46	100
Stefan	17.94	82.06	100
Mobile	19.01	80.99	100
Football	11.82	88.18	100
Salesman	14.56	85.44	100

**Table 3:** H.264 format calculation results.

Video camera	Resolution	kbps	Frames/s	MB/h	Hour	GB/day
1	CIF	110	5	49.5	8	0.4
2	CIF	250	15	112.5	8	0.9
3	4CIF	600	15	270	12	3.2

**Table 4:** MPEG-4 format calculation results.

Video camera	Resolution	Kbps	Frames/s	MB/h	Hour	GB/day
1	CIF	170	5	76.5	8	0.6
2	CIF	400	15	180	8	1.4
3	4CIF	880	15	396	12	5

**Table 5:** M.JPEG format calculation results.

Video camera	Resolution	kbps	Frames/s	MB/h	Hour	GB/day
1	CIF	13	5	234	8	1.9
2	CIF	13	15	702	8	5.6
3	4CIF	40	15	2160	12	26

## Data Availability

No data were used to support this study.
